The article "Biomarkers for Presymptomatic Doxorubicin-Induced Cardiotoxicity in Breast Cancer Patients" was retracted in 2019. Reason: lack of ethics approval or compliance.

# Biomarkers for Presymptomatic Doxorubicin-Induced Cardiotoxicity in Breast Cancer Patients

**DOI:** 10.1371/journal.pone.0160224

**Published:** 2016-08-04

**Authors:** Valentina K. Todorova, Issam Makhoul, Eric R. Siegel, Jeanne Wei, Annjanette Stone, Weleetka Carter, Marjorie L. Beggs, Aaron Owen, V. Suzanne Klimberg

**Affiliations:** 1 Department of Surgery/Breast Surgical Oncology, University of Arkansas for Medical Sciences, Little Rock, AR, United States of America; 2 Department of Hematology/Oncology, University of Arkansas for Medical Sciences, Little Rock, AR, United States of America; 3 Department of Biostatistics, University of Arkansas for Medical Sciences, Little Rock, AR, United States of America; 4 Department of Geriatrics, University of Arkansas for Medical Sciences, Little Rock, AR, United States of America; 5 Pharmacogenomics Analysis Laboratory, Research and Development Service, Central Arkansas Veterans Healthcare System, Little Rock, AR, United States of America; 6 Nephropath, Little Rock, AR, United States of America; University of North Carolina at Chapel Hill School of Medicine, UNITED STATES

## Abstract

Cardiotoxicity of doxorubicin (DOX) remains an important health concern. DOX cardiotoxicity is cumulative-dose-dependent and begins with the first dose of chemotherapy. No biomarker for presymptomatic detection of DOX cardiotoxicity has been validated. Our hypothesis is that peripheral blood cells (PBC) gene expression induced by the early doses of DOX-based chemotherapy could identify potential biomarkers for presymptomatic cardiotoxicity in cancer patients. PBC gene expression of 33 breast cancer patients was conducted before and after the first cycle of DOX-based chemotherapy. Cardiac function was evaluated before the start of chemotherapy and at its completion. Differentially expressed genes (DEG) of patients who developed DOX-associated cardiotoxicity after the completion of chemotherapy were compared with DEG of patients who did not. Ingenuity database was used for functional analysis of DEG. Sixty-sevens DEG (P<0.05) were identified in PBC of patients with DOX-cardiotoxicity. Most of DEG encode proteins secreted by activated neutrophils. The functional analysis of the DEG showed enrichment for immune- and inflammatory response. This is the first study to identify the PBC transcriptome signature associated with a single dose of DOX-based chemotherapy in cancer patients. We have shown that PBC transcriptome signature associated with one dose of DOX chemotherapy in breast cancer can predict later impairment of cardiac function. This finding may be of value in identifying patients at high or low risk for the development of DOX cardiotoxicity during the initial doses of chemotherapy and thus to avoid the accumulating toxic effects from the subsequent doses during treatment.

The article "Biomarkers for Presymptomatic Doxorubicin-Induced Cardiotoxicity in Breast Cancer Patients" was retracted in 2019. Reason: lack of ethics approval or compliance.

## Introduction

Doxorubicin (DOX), a commonly used anthracycline antibiotic for treatment of various malignancies may cause unpredictable cardiotoxicity [1]. DOX cardiotoxicity is cumulative-dose-dependent and begins with the first dose, suggesting that assessment of the cardiac function in patients at early doses of chemotherapy can avoid permanent cardiac damage [2]. According to the American College of Cardiology guidelines, patients receiving chemotherapy are at increased risk of developing cardiac dysfunction [3].

Evidence indicates that susceptibility to DOX cardiotoxicity is largely individual with some patients developing cardiomyopathy at doses of 200–400 mg/m^2^ [3], and others tolerating >1000 mg/m^2^ [4], suggesting the presence of a genetic predisposition.

Serial measurements of heart left ventricle ejection fraction (LVEF) is commonly used for cardiac monitoring during anthracycline treatment [5], although the prognostic value of LVEF appears to be controversial [6]. In some studies cardiotoxicity was defined as LVEF decrease by absolute 10% and/or to below 55% [7], in others cardiotoxicity was defined as a decrease below 45% [8]. A serious disadvantage of this test is the exposure to radioactivity along with the low predictability of pre-symptomatic cardiac damage [9]. Blood cardiac biomarkers, such as cardiac troponins and B-type natriuretic peptide (BNP) have been used in the diagnostics of heart failure [10], but other diseases have also been associated with increased troponin release [e.g. acute pulmonary embolism [11], and end-stage renal disease [12] and/or BNPs [e.g. end-stage renal disease [13]. Several studies failed to detect any correlation between concentrations of troponin and/or BNP and DOX-induced cardiotoxicity [14, 15].

Our previous study showed a high similarity between the gene expression of heart and peripheral blood cells (PBCs) in a rat model of DOX-cardiotoxicity [16], suggesting that PBC can be used as a surrogate tissue for assessing biomarkers of DOX cardiotoxicity. We hypothesize that PBC gene expression induced by the early doses of DOX-based chemotherapy could identify potential biomarkers for presymptomatic cardiotoxicity in cancer patients.

## Materials and Methods

### Study subjects and blood samples

Fifty-five women treated for breast cancer with DOX-based chemotherapy at the University of Arkansas for Medical Sciences were enrolled initially in an Institutional Review Board-approved protocol with written informed consent for each patient. All patients were treated with a predefined protocol which included a combination of DOX (Adriamycin, 60 mg/m^2^) with cyclophosphamide (600 mg/m^2^). However, 22 of these patients decided to dropout from the study for various reasons. We were able to obtain RNAs and data about cardiac function of 33 subjects.

The article "Biomarkers for Presymptomatic Doxorubicin-Induced Cardiotoxicity in Breast Cancer Patients" was retracted in 2019. Reason: lack of ethics approval or compliance.

Blood samples were collected prior to chemotherapy and after the first cycle of chemotherapy. PBCs were isolated from EDTA anti-coagulated blood using standard Ficoll-Paque Plus gradient centrifugation (density 1.073 g/mL) according to the instructions of the manufacturer (GE Healthcare, USA). Briefly, EDTA anti-coagulated blood, diluted with an equal volume of phosphate-buffered saline (PBS) was layered over the Ficoll-Paque Plus and was centrifuged at 400 g for 30 min at 18°C-20° with the brake off. After removing the upper layer containing plasma and platelets, the layer of peripheral blood mononuclear cells (PBMCs) was isolated and stored at -80° until further use. Total RNA was extracted from PBC using RNeasy columns (Qiagen; Valencia, CA) and samples with RNA integrity number (RIN) score>7 were used for expression analysis.

### Ethics Statement

This study was carried out in accordance with the ethical guidelines of the 1975 Declaration of Helsinki and was approved by the ethics committee of the University of Arkansas for Medical Sciences. All subjects signed an IRB approved informed consent where they were informed for the use of their blood samples and medical records for research purposes.

### Assessment of LVEF as a measure of cardiac function

Cardiac function of the patients was assessed by a multigated acquisition (MUGA) scan before the start of DOX- treatment and at its completion. A decline of LVEF by >10% or below 50% was considered abnormal [17].

### Microarray gene expression and data analysis

The gene expression screen was performed using HumanHT-12 v4 Expression BeadChip array (Illumina, San Diego, California). Raw data were further analyzed using Illumina GenomeStudio software.

PBC gene expression data were log2 –transformed and gene transcripts with average log2-intensities >7 were considered to be expressed. We first compared baseline levels of gene expression between the two groups of patients, and then examined expression changes from baseline to after the first cycle of chemotherapy in each group of patients. The group-specific means for each group (“abnormal MUGA scan” and “normal MUGA scan”) were analyzed via repeated-measures ANOVA for expression changes after DOX. Genes with p-value <0.05 were considered differentially expressed. To adjust for multiple testing, the Benjamini-Hochberg false discovery rate (FDR) was used [18]. Given our relatively small sample size, we chose to use a FDR corrected significance threshold P≤ 0.1 which is commonly used in hypothesis-generating, discovery-driven gene expression studies [19].

The article "Biomarkers for Presymptomatic Doxorubicin-Induced Cardiotoxicity in Breast Cancer Patients" was retracted in 2019. Reason: lack of ethics approval or compliance.

### Functional annotation

Functional network analysis was performed using Ingenuity Pathways Analysis System; http://www.ingenuity.com) which identifies the most significant biological functions to a dataset based on the causal relationships previously reported in the literature.

### QRT-PCR Validation

Quantitative real-time RT-PCR was used for evaluation and confirmation of the gene expression data. Total RNAs were reverse transcribed and cDNAs were amplified using Nugen Ovation RNA Amplification System V2 (NuGEN^™^ Technologies, San Carlos, CA). QPCR was performed using Taqman Universal Fast PCR master mix and specific primers for DEFA3, DEFA4, ELANE, ARG1, HP, CEACAM8, and 18S tRNA (Applied Biosystems, Foster City, CA). Data were analyzed using the 2-deltadelta Ct method. The Ct values of both the control and the samples of interest were normalized to 18S. DeltaCt was calculated as “deltaCt(gene) equals Ct(18S) minus Ct(gene)”. DOX response was calculated as deltaCt “After DOX” minus deltaCt “Before DOX”, and is in ddCt (delta-delta-Ct) units.

## Results

### Characteristics of study subjects

We have analyzed and compared PBC gene expression associated with one dose of DOX-based chemotherapy of 8 breast cancer patients who developed abnormal LVEF after the completion of chemotherapy and 25 breast cancer patients who did not. Patients’ characteristics are provided in Table 1.

**Table 1:** Cardiac function of women with breast cancer, treated with DOX-based chemotherapy. MUGA scan was performed before the start of DOX chemotherapy and at its completion.

	Number of patients	Average LVEF (%) at baseline*	Average LVEF (%) at completion of chemotherapy*
**Patients with abnormal LVEF (%)**	8	69.875 ± 5.436	57.875 ± 3.833
** 18–47 years**	2	68.5 ± 2.121	57.5 ± 0.707
** 48–55 years**	2	64.0 ± 0	54.0 ± 0
** >56 years**	4	73.5 ± 5.066	60.0 ± 4.242
**Patients with normal LVEF (%)**	25	61.583 ± 5.523	61.833 ± 6.919
** 18–47 years**	9	60.888 ± 6.050	62.222 ± 9.162
** 48–55 years**	9	60.888 ± 5.065	59.777 ± 5.118
** >56 years**	7	63.142 ± 5.080	57.714 ± 6.499

LVEF, left ventricle ejection fraction

*Mean ± SD

### Gene expression profile associated with a single dose of DOX-based chemotherapy

The volcano plots on Fig 1 show the probability that the gene is differentially expressed in a data of average ‘before vs. after’ one dose of DOX-based chemotherapy in all women (1A) and in the groups with normal (1B), and abnormal LVEF (1C). The analysis of the gene expression of PBC indicated that a single dose of DOX induced significant changes in the expression of 235 genes (fold change >1.5, FDR<0.1) (Table 2). There were no significant differences between the gene expression of the two groups of patients (abnormal and normal LVEF) at baselines (P>0.05, FDR>0.1).

The article "Biomarkers for Presymptomatic Doxorubicin-Induced Cardiotoxicity in Breast Cancer Patients" was retracted in 2019. Reason: lack of ethics approval or compliance.

**Table 2:** Differentially expressed genes in PBC of breast cancer patients after the 1^st^ cycle of DOX-based chemotherapy versus baseline (before the start of chemotherapy).

SYMBOL	Estimate*	P-value	FDR
**FAM129C**	-0.7106	<.0001	0.00149
**LOC283663**	-1.0472	<.0001	0.00149
**HLA-DOB**	-1.1215	<.0001	0.00149
**VPREB3**	-1.3445	<.0001	0.00149
**TCL1A**	-1.4775	<.0001	0.00149
**FCRLA**	-1.8054	<.0001	0.00171
**CD19**	-1.5499	<.0001	0.00196
**DEFA3**	3.7012	<.0001	0.00203
**LOC653600**	3.6557	<.0001	0.00203
**PGLYRP1**	3.396	<.0001	0.00203
**CEACAM8**	3.2916	<.0001	0.00203
**KIAA0367**	0.7253	<.0001	0.00203
**OSBPL10**	-0.9924	<.0001	0.00203
**LOC90925**	-1.0736	<.0001	0.00203
**CAMP**	3.2632	<.0001	0.00231
**DEFA1**	3.499	<.0001	0.00276
**DEFA1B**	3.3555	<.0001	0.00276
**MMP9**	3.287	<.0001	0.00276
**MMP8**	2.8754	<.0001	0.00276
**TFF3**	1.9749	<.0001	0.00276
**PROM1**	0.7141	<.0001	0.00276
**CRISP3**	1.3036	<.0001	0.00277
**HLA-DOA**	-0.7107	<.0001	0.0028
**TCN1**	3.052	<.0001	0.00331
**ELANE**	2.8036	<.0001	0.00331
**OLFM4**	2.7531	<.0001	0.00331
**ARG1**	2.6483	<.0001	0.00331
**HP**	2.6308	<.0001	0.00331
**CXCR5**	-0.907	<.0001	0.00331
**CEACAM6**	2.6645	<.0001	0.00336
**DEFA4**	2.9771	<.0001	0.00337
**ANXA3**	2.5028	<.0001	0.00348
**BPI**	2.5084	<.0001	0.00389
**OLR1**	2.3894	<.0001	0.00389
**S100P**	2.3653	<.0001	0.00414
**ORM1**	2.3809	<.0001	0.00486
**DLGAP5**	0.6505	<.0001	0.00488
**SPIB**	-0.6947	<.0001	0.00561
**MS4A3**	1.8872	<.0001	0.00598
**BANK1**	-0.6946	<.0001	0.00598
**CTSG**	2.3894	<.0001	0.00617
**FCER2**	-0.7478	<.0001	0.00617
**CEACAM1**	1.993	<.0001	0.00618
**SPTA1**	0.8716	<.0001	0.00618
**TNFAIP6**	0.7898	<.0001	0.00618
**LOC728014**	-0.6389	<.0001	0.00622
**CDC20**	0.7971	<.0001	0.00632
**IFIT1L**	2.2327	<.0001	0.00643
**HBM**	2.1896	<.0001	0.00643
**TRPM6**	0.6271	<.0001	0.00653
**GYPB**	1.3679	<.0001	0.00692
**DACH1**	0.6661	<.0001	0.00765
**LIN7A**	0.5931	<.0001	0.00765
**CD79A**	-1.6211	<.0001	0.00765
**ASPM**	0.6487	<.0001	0.00782
**LOC653061**	1.2216	<.0001	0.00849
**COBLL1**	-0.6696	<.0001	0.00858
**PTPN20**	1.1766	<.0001	0.00861
**FCRL3**	-0.5891	<.0001	0.00861
**CA1**	2.3957	<.0001	0.00884
**IFI27**	0.9104	<.0001	0.00884
**BEX1**	1.2861	<.0001	0.00944
**LTF**	2.6717	<.0001	0.00949
**MPO**	2	<.0001	0.00953
**EPB42**	1.7482	<.0001	0.00953
**CA4**	1.7017	<.0001	0.00953
**BPGM**	1.0836	<.0001	0.00953
**ORM2**	0.9493	<.0001	0.00953
**GYPE**	0.9377	<.0001	0.00953
**RAP1GAP**	1.1026	<.0001	0.00986
**CCNB2**	0.6868	<.0001	0.00986
**BIRC3**	-0.6637	<.0001	0.01018
**NCAPG**	0.5988	0.0001	0.01092
**SESN3**	0.8006	0.0001	0.01111
**RAB3IL1**	0.6721	0.0001	0.01111
**C5orf32**	1.4237	0.0001	0.0117
**SERPINB10**	1.1818	0.0001	0.0117
**COL17A1**	1.433	0.0001	0.0118
**BLK**	-0.6487	0.0001	0.01186
**RETN**	1.9094	0.0001	0.01241
**C6orf173**	0.5965	0.0001	0.0128
**C19orf59**	1.0429	0.0002	0.01297
**TSPAN2**	0.6938	0.0002	0.01297
**ANKRD22**	1.0776	0.0002	0.01306
**CDC45L**	0.6344	0.0002	0.01353
**RNASE3**	1.9597	0.0002	0.01361
**LOC643332**	1.0172	0.0002	0.01361
**NFIX**	0.7093	0.0002	0.01445
**SLC22A4**	0.732	0.0002	0.01464
**NUSAP1**	0.7046	0.0002	0.01466
**LOC651524**	1.0154	0.0002	0.01471
**FAR2**	1.1622	0.0002	0.01494
**RNF182**	0.6275	0.0002	0.01494
**CPA3**	0.697	0.0002	0.01608
**FECH**	0.8687	0.0002	0.01611
**ERCC5**	-0.6263	0.0003	0.01695
**CD79B**	-1.2326	0.0003	0.01703
**CEP55**	0.5971	0.0003	0.01732
**UIMC1**	-0.763	0.0003	0.01732
**CHI3L1**	1.3608	0.0003	0.01741
**CDA**	1.0502	0.0003	0.01783
**ATP8B4**	0.8687	0.0003	0.01836
**OSBP2**	1.1908	0.0003	0.01845
**LOC100134379**	1.5894	0.0003	0.01851
**ABCA13**	1.3413	0.0004	0.0193
**SLC22A16**	0.6917	0.0004	0.01962
**DYSF**	1.0349	0.0004	0.01989
**GPR84**	1.0967	0.0004	0.02007
**CYP4F3**	1.0235	0.0004	0.02117
**LOC283392**	0.7064	0.0004	0.02117
**VNN1**	0.6997	0.0004	0.02163
**LOC642103**	0.9778	0.0005	0.02428
**FCGR1A**	0.7202	0.0005	0.02439
**SELENBP1**	1.2147	0.0005	0.02454
**TACSTD2**	1.3185	0.0006	0.02542
**TYMS**	0.919	0.0006	0.02547
**HBE1**	0.714	0.0006	0.02547
**SLPI**	1.3417	0.0006	0.02675
**CLC**	1.3377	0.0006	0.0268
**CKAP4**	0.8558	0.0006	0.0268
**VAV1**	-0.6377	0.0006	0.0268
**RNASE2**	1.463	0.0006	0.02709
**CEBPE**	1.1338	0.0006	0.0271
**CEACAM3**	0.6023	0.0007	0.0273
**AHSP**	2.0537	0.0007	0.02786
**HMBS**	0.602	0.0007	0.02788
**RBM33**	-0.6091	0.0007	0.02844
**SLC27A2**	0.6294	0.0007	0.02855
**MANSC1**	0.6188	0.0008	0.02941
**TMCC2**	0.808	0.0008	0.02952
**ITPR3**	-0.797	0.0008	0.02975
**S100A12**	1.208	0.0008	0.02986
**MYB**	0.9609	0.0008	0.03063
**HBD**	2.0496	0.0008	0.03076
**GOLGA8B**	-0.856	0.0008	0.0309
**ALPL**	1.3904	0.0008	0.03113
**MGC42367**	0.6187	0.0008	0.03113
**LCN2**	2.2325	0.0008	0.03136
**STX3**	0.6528	0.0009	0.03263
**PLSCR1**	0.7974	0.0009	0.03323
**CLEC4D**	0.6695	0.0009	0.03382
**GADD45G**	0.6235	0.001	0.03449
**KRT1**	0.9562	0.001	0.03461
**CD24**	1.4399	0.001	0.0351
**BST1**	0.7232	0.001	0.03512
**PCOLCE2**	0.9448	0.0011	0.03573
**TOP2A**	0.697	0.0011	0.03615
**LOC440313**	0.6087	0.0012	0.0375
**B4GALT5**	0.9484	0.0012	0.03821
**NLRC4**	0.6716	0.0012	0.03859
**C1QB**	0.6326	0.0013	0.03971
**XK**	0.7828	0.0013	0.03989
**FSTL3**	0.607	0.0014	0.04028
**ABHD5**	0.6037	0.0015	0.04212
**PFKFB3**	0.7688	0.0015	0.04228
**CITED4**	0.6897	0.0015	0.04269
**PRC1**	0.6001	0.0015	0.04273
**QPCT**	0.8802	0.0016	0.04286
**CD177**	0.8838	0.0017	0.04393
**TFDP1**	0.6815	0.0019	0.04653
**TESC**	0.6841	0.0021	0.04934
**TMOD1**	0.7627	0.0022	0.05019
**FCGR1C**	0.5994	0.0022	0.05032
**HBG1**	2.077	0.0023	0.05116
**NPL**	0.5947	0.0023	0.05121
**FAIM3**	-0.7711	0.0023	0.05195
**LOC653778**	1.0179	0.0024	0.05256
**SCD**	0.6756	0.0024	0.05256
**LOC389599**	0.9621	0.0025	0.05334
**LRG1**	0.7248	0.0025	0.05334
**SLAMF6**	-0.7282	0.0025	0.05334
**EEF1D**	-0.7883	0.0026	0.05387
**C5AR1**	0.6534	0.0026	0.05407
**ZMAT3**	-0.7805	0.0026	0.05487
**TNS1**	0.6804	0.0028	0.05614
**BASP1**	0.7966	0.003	0.05803
**LRAP**	-1.0002	0.003	0.05857
**LOC100132391**	-1.1762	0.0031	0.05908
**HBG2**	2.0155	0.0032	0.0599
**LOC100129362**	-1.0645	0.0032	0.06051
**GPR160**	0.6186	0.0033	0.0611
**LRRFIP1**	-0.712	0.0034	0.06199
**ARL16**	-0.8601	0.0035	0.06261
**SAP30**	0.6245	0.0035	0.0627
**HK3**	0.6149	0.0035	0.06275
**RGL4**	1.0261	0.0035	0.06297
**SERPINA13**	0.6036	0.0036	0.06345
**E2F2**	0.832	0.0039	0.06504
**STMN3**	-0.709	0.0039	0.06506
**ALAS2**	1.4889	0.004	0.06583
**FPR2**	0.7452	0.0041	0.06685
**LOC441087**	-0.9447	0.0041	0.06685
**LOC728620**	-0.8585	0.0043	0.06822
**LOC100132499**	-0.7917	0.0044	0.06922
**MLLT6**	-0.711	0.0045	0.06996
**QRFPR**	-0.8583	0.0047	0.07174
**STRADB**	0.8962	0.0047	0.07192
**SLC2A5**	0.99	0.005	0.07341
**CREG1**	0.6149	0.0052	0.07511
**ZNF549**	-0.7673	0.0053	0.07601
**UGCG**	0.8707	0.0054	0.07686
**LOC728809**	-1.1654	0.0058	0.07957
**KRT72**	-0.6038	0.0059	0.07973
**DUSP19**	-1.0172	0.0059	0.07973
**TP53I13**	-0.5914	0.0059	0.08
**XPNPEP3**	-0.9484	0.0061	0.08109
**C14orf85**	-1.0189	0.0065	0.08295
**FLJ22662**	0.7316	0.0066	0.08321
**LOC654103**	0.9414	0.0071	0.08649
**GYG1**	0.6746	0.0072	0.08668
**CDKN2AIPNL**	-0.9848	0.0073	0.08745
**FCGR1B**	0.6819	0.0073	0.08753
**PLA2G4B**	-0.6336	0.0073	0.08753
**GCA**	0.8787	0.0074	0.08772
**BMS1P5**	-0.9416	0.0075	0.08887
**MOSC1**	0.5856	0.0078	0.09043
**IL7R**	-0.6069	0.0078	0.09095
**GBE1**	0.5874	0.0079	0.09142
**HSPC268**	-0.7923	0.0081	0.0917
**HMHA1**	-0.6014	0.0081	0.0917
**LOC728888**	-0.6524	0.0083	0.093
**SLC25A37**	0.8626	0.0085	0.09382
**LOC100133516**	-0.6214	0.0085	0.09412
**GPR175**	0.6802	0.0086	0.09427
**HCG2P7**	-0.9518	0.0087	0.09435
**CD27**	-0.7256	0.009	0.09578
**LOC100128288**	-0.8262	0.009	0.09603
**FAM175A**	-0.9464	0.0093	0.09751
**DUXAP3**	-0.808	0.0094	0.09823
**EID2B**	-0.8188	0.0094	0.09824
**DDX51**	-0.8393	0.0094	0.09824
**C3orf34**	-0.6914	0.0096	0.09932
**LOC100128084**	-1.0162	0.0097	0.09932
**CD6**	-0.7416	0.0097	0.09945
**LMOD3**	-0.7242	0.0097	0.09947

*log2 fold change

The article "Biomarkers for Presymptomatic Doxorubicin-Induced Cardiotoxicity in Breast Cancer Patients" was retracted in 2019. Reason: lack of ethics approval or compliance.

**Fig 1:** Volcano plots of log2 fold change (x-axis) versus –log10 of unadjusted P-values (y-axis), representing the probability that the gene is differentially expressed in PBC of breast cancer patients treated with DOX-based chemotherapy in data of average before versus after one dose of DOX-based chemotherapy. (A) comparison of average before vs after of all patients; (B) average before vs after in patients with normal LVEF after the completion of chemotherapy; (C) average before vs after in patients with abnormal LVEF after the completion of chemotherapy. P<0.05; FDR<0.1.

We have also compared the gene expression of the 33 patients divided into 3 age groups, each comprising 11 patients, 18–47 years (youngest), 48–55 years (mid-age) and 56–99 years (oldest). A single dose of DOX-based chemotherapy resulted in 66 differentially expressed genes (DEG) with log2 fold change (FC)>1.0 (p<0.05, FDR<0.05) in the oldest group of patients in comparison with the other two age-groups (Table 3).

**Table 3:** Age-associated differences in the gene expression.

Symbol	56–99 years*#	48–55 years*	18–47 years*
**MMP9**	3.9123	1.2884	3.033
**PGLYRP1**	3.8371	1.4919	3.293
**CEACAM8**	3.5834	1.4616	2.977
**MMP8**	3.5284	1.5207	2.002
**TCN1**	3.4311	1.0817	2.783
**LTF**	3.4051	1.0024	2.083
**DEFA4**	3.3439	1.2729	2.607
**HP**	3.3082	1.1380	1.977
**ELANE**	3.2522	1.1366	2.541
**ARG1**	3.2388	1.2595	1.874
**CEACAM6**	3.1734	1.3527	2.143
**OLFM4**	3.1396	1.4073	2.447
**ANXA3**	3.1026	1.5605	1.846
**BPI**	3.0445	0.9567	2.189
**OLR1**	2.9252	1.1325	1.825
**S100P**	2.9251	1.1516	1.996
**ORM1**	2.8422	1.1065	1.895
**CTSG**	2.8168	0.9180	2.038
**RNASE3**	2.6924	0.8301	1.138
**RETN**	2.6141	0.6415	1.574
**CEACAM1**	2.5762	1.0244	1.238
**MPO**	2.5563	0.8955	1.358
**TFF3**	2.3798	0.9370	1.590
**MS4A3**	2.3296	0.6207	1.363
**CA4**	2.2531	0.7716	1.039
**ALPL**	2.1398	0.2850	1.074
**ABCA13**	1.9824	0.7552	0.577
**COL17A1**	1.9809	0.6801	0.833
**C5orf32**	1.9765	0.5603	0.833
**CHI3L1**	1.9577	0.6048	0.743
**SLPI**	1.9103	0.6521	0.746
**CEBPE**	1.7418	0.4987	0.524
**SERPINB10**	1.7352	0.4157	0.778
**BEX1**	1.7131	0.7104	0.891
**FAR2**	1.6847	0.4184	0.567
**GPR84**	1.6349	0.4278	0.469
**CDA**	1.5593	0.1996	0.724
**CYP4F3**	1.5434	0.4521	0.487
**UGCG**	1.5267	0.3211	0.364
**DYSF**	1.5088	0.2250	0.641
**CRISP3**	1.4774	0.8383	0.942
**PCOLCE2**	1.4609	0.4807	0.493
**PTPN20**	1.4439	0.5310	0.875
**B4GALT5**	1.4165	0.3049	0.641
**TYMS**	1.4060	0.3998	0.423
**ORM2**	1.3950	0.3985	0.524
**CD177**	1.3648	0.3258	0.366
**CKAP4**	1.2778	0.3066	0.594
**ATP8B4**	1.2184	0.4067	0.423
**LRG1**	1.2139	0.0939	0.398
**VNN1**	1.1638	0.2104	0.195
**BST1**	1.1578	0.2298	0.325
**TNFAIP6**	1.1326	0.2886	0.406
**CITED4**	1.1228	0.2629	0.353
**GPR160**	1.0819	0.1431	0.098
**SCD**	1.0804	0.2424	0.225
**SLC22A16**	1.0467	0.3010	0.398
**STX3**	1.0319	0.3519	0.231
**MANSC1**	1.0227	0.1727	0.238
**CLEC4D**	1.0037	0.1743	0.204
**ADARB1**	-0.5014	-0.2387	-0.351
**HLA-DOB**	-1.2817	-0.5855	-0.931
**VPREB3**	-1.4604	-0.9855	-1.053
**TCL1A**	-1.4833	-1.3079	-1.210
**CD19**	-1.7652	-1.0990	-1.258
**FCRLA**	-2.1067	-1.2568	-1.254

*Log2 fold change

^#^ p<0.05, FDR<0.05

The article "Biomarkers for Presymptomatic Doxorubicin-Induced Cardiotoxicity in Breast Cancer Patients" was retracted in 2019. Reason: lack of ethics approval or compliance.

### Gene expression profile in patients with abnormal decline of LVEF

The analysis of the expression profiling of PBC after one dose of DOX-based chemotherapy in women who developed abnormal LVEF after a full course of chemotherapy found 80 transcripts that differed >1.5-fold (p<0.05, FDR<0.1) from the baseline, 13 of which were shared with women with normal LVEF. Table 4 shows the unique DEG in patients with abnormal LVEF.

**Table 4:** Unique DOX-induced DEG in patients with abnormal decline of LVEF after one dose of DOX-based chemotherapy (p<0.05, FDR<0.1).

SYMBOL	Log 2 FC*	GENE ID	DESCRIPTION
**DEFA3**	5.14	HGNC = 2762|UniProtKB = P59666	Neutrophil defensin 3;DEFA3
**DEFA1**	4.96	HGNC = 33596|UniProtKB = P59665	Neutrophil defensin 1;DEFA1
**CEACAM8**	4.49	HGNC = 1820|UniProtKB = P31997	Carcinoembryonic antigen-related cell adhesion molecule 8
**CAMP**	4.41	HGNC = 1472|UniProtKB = P49913	Cathelicidin antimicrobial peptide;CAMP;ortholog
**TCN1**	4.26	HGNC = 11652|UniProtKB = P20061	Transcobalamin-1;TCN1;ortholog
**DEFA4**	4.08	HGNC = 2763|UniProtKB = P12838	Neutrophil defensin 4;DEFA4;ortholog
**MMP8**	3.89	HGNC = 7175|UniProtKB = P22894	Neutrophil collagenase;MMP8;ortholog
**ELANE**	3.76	HGNC = 3309|UniProtKB = P08246	Neutrophil elastase;ELANE;ortholog
**ARG1**	3.67	HGNC = 663|UniProtKB = P05089	Arginase-1;ARG1;ortholog
**HP**	3.58	HGNC = 5141|UniProtKB = P00738	Haptoglobin;HP;ortholog
**CEACAM6**	3.52	HGNC = 1818|UniProtKB = P40199	Carcinoembryonic antigen-related cell adhesion molecule 6
**BPI**	3.37	HGNC = 1095|UniProtKB = P17213	Bactericidal permeability-increasing protein;BPI;ortholog
**CTSG**	3.29	HGNC = 2532|UniProtKB = P08311	Cathepsin G;CTSG;ortholog
**OLR1**	3.22	HGNC = 8133|UniProtKB = P78380	Oxidized low-density lipoprotein receptor 1;OLR1;ortholog
**ORM1**	3.22	HGNC = 8498|UniProtKB = P02763	Alpha-1-acid glycoprotein 1;ORM1;ortholog
**S100P**	3.03	HGNC = 10504|UniProtKB = P25815	Protein S100-P;S100P;ortholog
**MS4A3**	2.76	HGNC = 7317|UniProtKB = Q96HJ5	Membrane-spanning 4-domains subfamily A member 3
**CEACAM1**	2.73	HGNC = 1814|UniProtKB = P13688	Carcinoembryonic antigen-related cell adhesion molecule 1
**TFF3**	2.63	HGNC = 11757|UniProtKB = Q07654	Trefoil factor 3;TFF3;ortholog
**CLC**	2.45	HGNC = 2014|UniProtKB = Q05315	Galectin-10;CLC;ortholog
**GYPB**	1.99	HGNC = 4703|UniProtKB = P06028	Glycophorin-B;GYPB;ortholog
**CRISP3**	1.73	HGNC = 16904|UniProtKB = P54108	Cysteine-rich secretory protein 3;CRISP3;ortholog
**RAP1GAP**	1.69	HGNC = 9858|UniProtKB = P47736	Rap1 GTPase-activating protein 1;RAP1GAP;ortholog
**ANKRD22**	1.64	HGNC = 28321|UniProtKB = Q5VYY1	Ankyrin repeat domain-containing protein 22;ANKRD22
**BPGM**	1.55	HGNC = 1093|UniProtKB = P07738	Bisphosphoglycerate mutase;BPGM;ortholog
**GYPE**	1.44	HGNC = 4705|UniProtKB = P15421	Glycophorin-E;GYPE;ortholog
**IFI27**	1.42	HGNC = 5397|UniProtKB = P40305	Interferon alpha-inducible protein 27, mitochondrial;IFI27
**FECH**	1.35	HGNC = 3647|UniProtKB = P22830	Ferrochelatase, mitochondrial;FECH;ortholog
**SPTA1**	1.29	HGNC = 11272|UniProtKB = P02549	Spectrin alpha chain, erythrocytic 1;SPTA1;ortholog
**CPA3**	1.27	HGNC = 2298|UniProtKB = P15088	Mast cell carboxypeptidase A;CPA3;ortholog
**SESN3**	1.20	HGNC = 23060|UniProtKB = P58005	Sestrin-3;SESN3;ortholog
**NFIX**	1.18	HGNC = 7788|UniProtKB = Q14938	Nuclear factor 1 X-type;NFIX;ortholog
**TNFAIP6**	1.14	HGNC = 11898|UniProtKB = P98066	Tumor necrosis factor-inducible gene 6 protein;TNFAIP6
**SLC22A4**	1.12	HGNC = 10968|UniProtKB = Q9H015	Solute carrier family 22 member 4;SLC22A4;ortholog
**CDC20**	1.10	HGNC = 1723|UniProtKB = Q12834	Cell division cycle protein 20 homolog;CDC20;ortholog
**KIAA0367**	1.10	HGNC = 25209|UniProtKB = Q8WUY3	Protein prune homolog 2;PRUNE2;ortholog
**RAB3IL1**	0.98	HGNC = 9780|UniProtKB = Q8TBN0	Guanine nucleotide exchange factor for Rab-3A;RAB3IL1;ortholog
**PROM1**	0.98	HGNC = 9454|UniProtKB = O43490	Prominin-1;PROM1;ortholog
**C6orf173**	0.93	HGNC = 21488|UniProtKB = O5EE01	C6orf173 protein;C6orf173;ortholog
**TRPM6**	0.93	HGNC = 17995|UniProtKB = Q9BX84	Transient receptor potential cation channel subfamily M member 6
**DACH1**	0.92	HGNC = 2663|UniProtKB = Q9UI36	Dachshund homolog 1;DACH1;ortholog
**ITLN1**	0.87	HGNC = 18259|UniProtKB = Q8WWA0	Intelectin-1;ITLN1;ortholog
**GYPA**	0.85	HGNC = 4702|UniProtKB = P02724	Glycophorin-A;GYPA;ortholog
**DLGAP5**	0.85	HGNC = 16864|UniProtKB = Q15398	Disks large-associated protein 5;DLGAP5;ortholog
**SERPINB2**	0.85	HGNC = 8584|UniProtKB = P05120	Plasminogen activator inhibitor 2;SERPINB2;ortholog
**RHAG**	0.83	HGNC = 10006|UniProtKB = Q02094	Ammonium transporter Rh type A;RHAG;ortholog
**LIN7A**	0.82	HGNC = 17787|UniProtKB = O14910	Protein lin-7 homolog A;LIN7A;ortholog
**TFDP2**	0.81	HGNC = 11751|UniProtKB = Q14188	Transcription factor Dp-2;TFDP2;ortholog
**HMMR**	0.75	HGNC = 5012|UniProtKB = O75330	Hyaluronan mediated motility receptor;HMMR;ortholog
**TGM2**	0.71	HGNC = 11778|UniProtKB = P21980	Protein-glutamine gamma-glutamyltransferase 2;TGM2;ortholog
**CKS2**	0.70	HGNC = 2000|UniProtKB = P33552	Cyclin-dependent kinases regulatory subunit 2;CKS2
**PRSSL1**	0.68	HGNC = 31397|UniProtKB = Q6UWY2	Uncharacterized protein;PRSSL1;ortholog
**PTTG1**	0.64	HGNC = 9690|UniProtKB = O95997	Securin;PTTG1;ortholog
**CD34**	0.63	HGNC = 1662|UniProtKB = P28906	Hematopoietic progenitor cell antigen CD34;CD34;ortholog
**PTRF**	0.63	HGNC = 9688|UniProtKB = Q6NZI2	Polymerase I and transcript release factor;PTRF;ortholog
**UBE2W**	0.60	HGNC = 25616|UniProtKB = Q96B02	Ubiquitin-conjugating enzyme E2 W;UBE2W;ortholog
**PRG2**	0.59	HGNC = 9362|UniProtKB = P13727	Bone marrow proteoglycan;PRG2;ortholog
**ZNF783**	-0.59	HGNC = 27222|UniProtKB = Q6ZMS7	Protein ZNF783;ZNF783;ortholog
**ZNF33B**	-0.64	HGNC = 13097|UniProtKB = Q06732	Zinc finger protein 33B;ZNF33B;ortholog
**C13orf18**	-0.65	HGNC = 20420UniProtKB = Q9H714	Uncharacterized protein KIAA0226-like
**CD72**	-0.67	HGNC = 1696|UniProtKB = P21854	B-cell differentiation antigen CD72;CD72;ortholog
**CD1C**	-0.68	HGNC = 1636|UniProtKB = P29017	T-cell surface glycoprotein CD1c;CD1C;ortholog
**GNG7**	-0.69	HGNC = 4410|UniProtKB = O60262	Guanine nucleotide-binding protein G(I)/G(S)/G(O) subunit gamma-7
**ZNF263**	-0.70	HGNC = 13056|UniProtKB = O14978	Zinc finger protein 263;ZNF263;ortholog
**SEL1L3**	-0.75	HGNC = 29108|UniProtKB = Q68CR1	Protein sel-1 homolog 3;SEL1L3;ortholog
**HLA-DOA**	-0.91	HGNC = 4936|UniProtKB = P06340	HLA class II histocompatibility antigen, DO alpha chain
**BANK1**	-0.93	HGNC = 18233|UniProtKB = Q8NDB2	B-cell scaffold protein with ankyrin repeats

*Log2 FC, Log2 fold change

Downregulation of TCL1A and FCRL was reported in breast cancer patients treated with several doses of DOX-based chemotherapy who developed cardiomyopathy [20]. Downregulation of CXCR5, which encodes chemokine expressed on B-cells could be explained with the depletion of B-cells in cancer patients treated with DOX-based chemotherapy [21, 22]. Lower expression of CD72 was detected in patients with systemic lupus erythematosus (SLE) and it correlated inversely with SLE disease activity [23].

The article "Biomarkers for Presymptomatic Doxorubicin-Induced Cardiotoxicity in Breast Cancer Patients" was retracted in 2019. Reason: lack of ethics approval or compliance.

The top upregulated DEG in the “abnormal” dataset were genes encoding the alpha-defensins DEFA1-4 (HNP-1 to -4), which are secreted by activated neutrophils and are involved in involved in innate immune response [24]. Significantly upregulated were several other genes encoding proteins secreted by activated neutrophils and associated with inflammation, such as BPI (bactericidal permeability increasing protein), ELANE (neutrophil elastase), CTSG (neutrophil cathepsin) [25,26]. ARG1 [27] which encodes arginase and HP which encodes haptoglobin [28] are involved in a variety of inflammatory diseases.The protein encoded by TNFAIP6 (tumor necrosis factor, alpha-induced protein 6) was found to be increased in the synovial fluid of patients with osteoarthritis and rheumatoid arthritis [29].

The 67 uniquely altered DEG in the group of patients with abnormal decline of LVEF was analyzed using Ingenuity software. The most enriched “biological functions” of this dataset identified using Ingenuity software were “cell-to-cell signaling” (p-value = 1.40E-07–3.2E-02), “cellular movement” (p value = 2.23E-04–2.02E-02) and “cellular development” (p value = 2.85E-04–2.89E-03) (Fig 2). In this category there were 8 molecules associated with “free radical scavenging” (p value = 8.26E-05–1.38E-03), which was expected, because one of the major mechanisms of DOX cardiotoxicity is oxidative damage. The most represented “diseases and disorders” were “connective tissue disorders” (p value 2.53E-12–2.57E-02), “inflammatory diseases” (p value = 2.53E-12–3.13E-02), “skeletal and muscular disorders” (2.53E-12–1.23E-02) and “immunological diseases” (p value = 5.59E-12–3.12E-02). Based on the curated literature data, an overlapping enrichment of molecules were identified in all of the top disease categories for rheumatic disease (RD), rheumatic arthritis (RA), SLE and infectious diseases. Multiple linked signaling pathways enriched for genes known to be involved primarily in inflammation and immunity were identified by Ingenuity in network 1 “Connective tissue disorder, Immunological disease, Inflammatory disease” which had 4 central nodes—NFKB, p38, ERK1/2 and AKT, all predicted to be upregulated (Fig 3A). The central nodes in network 2 “Cellular movement, Hematological system development and function, Immune cell trafficking” were IFN-gamma, TGFB, ARG1 and IL-4 (Fig 3B).

**Fig 2:** Ingenuity biological function analysis of DEG associated with 1 dose of DOX-based chemotherapy in patients with abnormal decline of LVEF at completion of chemotherapy. The most enriched “biological functions” of this dataset identified using Ingenuity software were “cell-to-cell signaling” (p-value = 1.40E-07–3.2E-02), “cellular movement” (p value = 2.23E-04–2.02E-02) and “cellular development” (p value = 2.85E-04–2.89E-03). The most represented “diseases and disorders” were “connective tissue disorders” (p value 2.53E-12–2.57E-02), “inflammatory diseases” (p value = 2.53E-12–3.13E-02), “skeletal and muscular disorders” (2.53E-12–1.23E-02) and “immunological diseases” (p value = 5.59E-12–3.12E-02).

The article "Biomarkers for Presymptomatic Doxorubicin-Induced Cardiotoxicity in Breast Cancer Patients" was retracted in 2019. Reason: lack of ethics approval or compliance.

**Fig 3:** Top interaction networks for the 67 DEG in PBC of patients with abnormal decline of LVEF after DOX-chemotherapy identified by Ingenuity pathway analysis. (A) Network 1 “Connective tissue disorder, Immunological disease, Inflammatory disease”; (B) Network 2 “Cellular movement, Hematological system development and function, Immune cell trafficking”. Red filled (up-regulation) and Green filled (down-regulation); Blue line (leads to inhibition); Orange line (leads to activation); Black line (effect not predicted).

### QRT-PCR Validation

The results (Table 5) from QRT-PCR confirmed the upregulation of the selected genes in patients with abnormal LVEF in comparison with the patients with normal LVEF.

**Table 5:** Results from QPCR of the target genes in breast cancer patients treated with DOX-based chempotherapy who developed abnromal decline in LVEF after the completion of chemotherapy.

Genes	Response differences ΔΔCt Units	95% Lower confidence limit	95% Upper confidence limit	P value	Fold change	Log2 fold change array data
**ARG1**	10.53	1.802	19.267	0.018	1483.1	3.6659
**CEACAM8**	20.92	5.154	36.687	0.0093	1984332	4.4908
**DEFA4**	16.312	6.135	26.489	0.0017	81350	4.0818
**DEFA3**	8.263	3.915	12.61	0.0002	307.126	5.137
**ELANE**	20.309	-3.113	43.73	0.0892	129871	3.762
**HP**	7.154	-0.257	14.564	0.0585	142.382	3.5814
**MMP9**	6.528	-2.515	15.57	0.1571	92.27	4.3398
**OLFM4**	37.053	-10.556	84.662	0.1272	1.43E+11	3.5721

## Discussion

DOX-based chemotherapy has greatly increased the number of long-term cancer survivors but has also led to an increasing number of patients experiencing DOX-induced cardiotoxicity [30]. Because there are no clinical methods for early detection of subclinical DOX cardiotoxicity, attempts to minimize cardiotoxicity include empiric DOX dose limitation or modification by risk factors, which pose a risk of premature discontinuation of effective anthracycline therapy. In addition, because of a wide individual variability in toxic anthracycline doses [31,32] cardiotoxicity may occur at unexpectedly low doses.

This is the first study to identify the PBC transcriptome signature associated with a single dose of DOX-based chemotherapy in cancer patients. We have identified a transcriptome signature associated with one dose of DOX-based chemotherapy which distinguished patients developing abnormal cardiac function after a full course of chemotherapy from those who maintained normal cardiac function. In addition, we have identified a gene expression profile associated with a single dose of DOX-based chemotherapy which distinguished older than younger patients.

As PBC are a subset of white blood cells, it is not surprising that the immune system was identified as the first and the most affected responder to the systemic stress of DOX-based chemotherapy. It has been found that the hyper-activated innate immune responses, including cytokine production, augmentation of natural killer (NK) cell activity [33], stimulation of cytotoxic T-lymphocyte (CTL) responses and augmentation of macrophages differentiation [34], could contribute to the progression of congestive heart failure. The top most significantly upregulated genes in the group of patients with abnormal LVEF decline encode proteins secreted by activated neutrophils, such as alpha-defensins, cathelicidins, arginase, cathepsin G, elastase and haptoglobin. Neutrophils provide the first line of innate immunity and are the major effectors of inflammation associated with cardiovascular diseases [35,36]. Several reports suggested the prognostic value of alpha-defensins [37], cathepsin G [38] and arginase [39] in heart failure. Our results indicate that there is a correlation between the severity of DOX-associated cardiotoxicity and the levels of activated neutrophils in the PBMC fraction of peripheral blood of breast cancer patients. The presence of abnormal subset of low density neutrophils in PBMC preparations have been reported in a range of conditions such as systemic lupus erythematosus (SLE), rheumatoid arthritis (RA) and acute rheumatic fever [40,41], cancer [42–45], vasculitis [46] and asthma [47], and their presence was correlated with disease activity. Several distinct features were identified in the low density neutrophils, such as different nuclear morphology, enhanced capacity to synthesize IFN I upon stimulation, higher expression of TNF-alpha, IL-6 and IL-8, and enhanced capacity to form neutrophil extracellular traps (NETs) [48,49]. NETs are characterized as chromatin fibers associated to granular proteins that are released to the extracellular space in order to immobilize and kill invading microbes during a process of cell death termed “NETosis” [50,51]. In addition to their antimicrobial role, recent evidence suggests that NETs can induce endothelial damage [52,53]. Denny et al [54] characterized the phenotype of low density neutrophil subset in SLE patients and found that the low density neutrophils displayed an impairment in the phagocytic potential, had proinflammatory phenotype and induced vascular damage, indicating that they contribute to accelerated atherosclerosis and cardiovascular disorders observed in SLE patients.

The article "Biomarkers for Presymptomatic Doxorubicin-Induced Cardiotoxicity in Breast Cancer Patients" was retracted in 2019. Reason: lack of ethics approval or compliance.

Because age-associated changes in DOX-induced gene expression has not been reported, we have compared the gene expression of the 33 patients divided into 3 age groups, 18–47 years (youngest), 48–55 years (mid-age), and 56–99 years (oldest). The results showed that a single dose of DOX-based chemotherapy resulted in 66 DEG in the oldest group of patients in comparison with the other two age-groups

The functional analysis of DEG in PBC of the subjects with abnormal cardiac function identified several linked pathways enriched for genes involved in inflammation and immunity and interconnected with NFKB, p38, ERK1/2, AKT, IFN-gamma, TGFB, ARG1 and IL-4, which were associated with ischemia [55], cardiac hypertrophy [56] and chronic heart failure [57]. Consistent with these reports, we found an overlapping enrichment of molecules for chronic inflammatory disorder, rheumatic arthritis, systemic lupus erythematosus and systemic autoimmune syndrome.

In conclusion, the results from this study show for the first-time that: 1) PBC transcriptome signature associated with early doses of DOX-based chemotherapy has the potential to predict later impairment of cardiac function and can be used as a surrogate marker for DOX-induced cardiotoxicity, 2) individual sensitivity to a single low dose of DOX is associated with differential expression of several genes implicated in inflammatory response and immune trafficking; 3) there is an overlapping but distinctive age-related pattern of gene expression associated with a single dose of DOX-based chemotherapy.

This finding may be of value in identifying patients at high or low risk for the development of DOX cardiotoxicity during the initial doses of chemotherapy and thus to avoid the accumulating toxic effects from the subsequent doses during treatment.
